# Prognosis Model of Advanced Non-Small-Cell Lung Cancer Based on Max-Min Hill-Climbing Algorithm

**DOI:** 10.1155/2022/9173913

**Published:** 2022-03-25

**Authors:** Weizheng Fu, Qingsheng Kan, Bin Li, Xiaoming Zhang

**Affiliations:** ^1^Department of Oncology, Suzhou Hospital of Anhui Medical University (Suzhou Municipal Hospital of Anhui Province), Suzhou 215002, China; ^2^Department of Radiology, Suzhou Hospital of Anhui Medical University (Suzhou Municipal Hospital of Anhui Province), Suzhou 215002, China; ^3^School of Basic Medical Sciences, Anhui Medical University, Hefei 230032, China

## Abstract

A safer and more effective treatment is need for the comprehensive treatment based on chemotherapy in patients with advanced non-small-cell lung cancer (NSCLC). The max-min hill-climbing (MMHC) is a common algorithm for disease prediction. This study is aimed at analyzing the efficacy of the MMHC algorithm in prognosis evaluation of advanced NSCLC. In this study, the prognosis model of lung cancer was first established by the MMHC algorithm. Then, according to the MMHC algorithm results, 40 patients with advanced NSCLC were divided into the research group and control group before anlotinib hydrochloride capsule combined with pemetrexed disodium chemotherapy. The diameter of solid tumor lesions, objective response rate (ORR), disease control rate (DCR), and progression-free survival (PFS) was compared between the two groups. The results showed that the MMHC model has a higher prediction accuracy of survival status of lung cancer patients. Under the guidance of the model, the research group has a smaller diameter of primary foci and metastatic foci, a higher ORR, DCR, and a longer PFS than the control group (*P* < 0.05). We can conclude that the MMHC algorithm can guide the maintenance treatment of advanced NSCLC, which is conducive to the prognosis judgment and treatment cost control.

## 1. Introduction

Lung cancer is a tumor with a very high degree of malignancy in clinical practice. Its mortality ranks the first among malignant tumors, and its incidence tends to rise year by year [1]. The non-small-cell lung cancer (NSCLC) accounts for more than 80% of all lung cancer patients, and about 50% of these patients have progressed to stage IIIB or IIIC at the time of treatment and have lost the best opportunity for surgery [2, 3].

At present, the clinical treatment of this disease mainly adopts the comprehensive treatment method based on chemotherapy. However, the effective rate of chemotherapy in most advanced NSCLC patients is very low, with the highest rate being only 20%-40% [4, 5]. Finding a safer and more effective treatment has become a hot topic in this field. Pemetrexed is often used to treat NSCLC clinically, with good therapeutic effect and less toxic and side effects [6]. In recent years, as a new tumor treatment method, molecular targeted therapy has been increasingly favored by doctors and patients. The drug inhibits the growth of tumor cells by precisely locating the carcinogenic sites [7]. Anlotinib is a new drug for targeted molecular therapy [8], but its safety and effectiveness remain to be further studied. If the prognosis of patients is poor, molecular targeted therapy cannot produce economic benefits. Therefore, it is of great significance to establish a predictive model suitable for clinical practice and considering multiple factors.

With the application of data mining technology in medical research, many scholars use machine learning methods for disease research [9–12]. Kim et al. [13] used the support vector machine to predict the 5-year survival of breast cancer patients. Chen et al. [14] used artificial neural network to establish the survival risk model of patients with NSCLC in four medical institutions. The max-min hill-climbing (MMHC) is a classical Bayesian network structure learning algorithm proposed by Tsamartinos in 2006 [15]. This algorithm is a local optimization method and an improvement of depth first search. It uses feedback information to help generate solution decisions. In this study, we first established the prediction model by MMHC in previous case data. Then, the effects of 40 patients with advanced NSCLC who came to our hospital were predicted by the model. Finally, the actual curative effect was analyzed.

## 2. Materials and Methods

### 2.1. General Information

The previous data set was selected from the lung cancer patients diagnosed in our hospital in the recent five years. The prognosis model was built by the maximum and minimum hill-climbing algorithm (MMHC). A total of 40 patients with advanced NSCLC in our hospital from January 2019 to July 2020 were selected as the validate database. According to the prediction results of the MMHC model, the patients were divided into the research group and control group. The study was approved by the hospital ethics committee, and informed consent was obtained from patients and their families.

### 2.2. Inclusion and Exclusion Criteria

Inclusion criteria were as follows: (1) the histologic examination diagnosed with NSCLC and patients clinical staging for III B or above, (2) over 18 years of age, (3) patients with a performance status score of 0-2 according to the physical condition established by the Eastern American Cancer Society group, (4) with measurable lesions and the expected survival time is more than three months, (5) epidermal growth factor receptor (EGFR) or anaplastic lymphoma kinase- (ALK-) positive in enrolled patients, and (6) all subjects gave informed consent and signed informed consent.

Exclusion criteria were as follows: (1) patients with primary tumors other than lung cancer; (2) patients with severe heart, liver, kidney, and other organ dysfunction; (3) patients suffering from neuropsychiatric diseases and unable to cooperate with this study; (4) the tumor has invaded essential blood vessels or during the follow-up treatment is likely to have massive bleeding patients; (5) women during pregnancy or lactation; (6) patients with deep venous thrombosis or pulmonary embolism; and (7) patients with other diseases were seriously endangering the life safety of patients or affecting the conduct of this study.

### 2.3. Establishment of Prognosis Model of Lung Cancer

#### 2.3.1. Feature Selection

According to tumor information and prognostic factors related to survival, 16 information variables including these factors were derived from the database: gender, marital status, location, affected side, pathological type, histological grading, tumor staging, degree of transfer, degree of diffusion, degree of lymph node accumulation, type of operation, radiotherapy or not, age of diagnosis, tumor size, number of lymph nodes, and examined number of positive lymph nodes. The last four variables were continuous, and the rest were discrete variables.

To improve the model's accuracy, the valuable features were selected from the above 16 information variables. Firstly, the chi-square test was passed in 12 variables (*P* < 0.05), which were marital status, histological grade, tumor stage, degree of metastasis, degree of diffusion, degree of lymph node accumulation, type of operation, radiotherapy or not, age of diagnosis, tumor size, number of lymph nodes examined, and positive number of lymph nodes. Then, the logistic regression analysis was used to filter the final characteristic variables. They were histological grade, tumor stage, diagnosis age, tumor size, number of examined lymph nodes, and number of positive lymph nodes. The screening results were shown in Table 1.

#### 2.3.2. Data Discretization

Both the final choice characteristic variables were are continuous data. These data should be discretized by the equidistant method. The main idea of this study is let the value range of continuous variable *X* be [*X*_min_, *X*_max_] and give the separable interval number “*r*” according to the prior knowledge. Since each interval is of equal width, the width of each interval is *d* = *X*_max_ − *X*_min_/*r*. The value *X*_*i*_ of continuous variable *X* and discrete level *j* (0 ≤ *j* ≤ *r* − 1) satisfies the following equation:

(1) $$\begin{array}{c} \left\{X_{i}=X_{\min},{\text{X}}_{\min}+\text{j}\times \text{d}<{\text{X}}_{\text{i}}\leq X_{\min}+\left(j+1\right)\times d,X_{i}=j+1\;X_{i}=0\right.. \end{array}$$

#### 2.3.3. Modeling Method

In disease survival prediction, the traditional statistical model is challenging to calculate the posterior probability and cannot directly express the relationship between variables. In this study, the Bayesian network method was used to establish the prognosis model of lung cancer. Bayesian network is a directed acyclic graph with parameters, which is represented by two tuples (*G*, *Θ*), where *G* = (*V*, *E*) is the directed acyclic graph of node relationship, which is called Bayesian network structure. Node set *V* = {*X*_1_, *X*_2_, ⋯, *X*_*n*_} is the random vector, and directed edge set *E* = {*e*_*ij*_ | *X*_*i*_⟶*X*_*j*_, *i*, *j* = 1, 2, ⋯, *n*} is the dependence between variables. Θ = {Θ_1_, Θ_2_, ⋯, Θ_*n*_} represents the conditional probability of node *X*_*i*_, which is called Bayesian network parameter. The parameter *o* of node *X* represents the conditional probability distribution of itself and its parent node set Pa(*X*_*i*_), which is Θ = P(*X*_*i*_ | *Pa*(*X*_*i*_)). In addition, any given Bayesian network satisfies the Markov condition; that is, ∀*X*_*i*_ ∈ *V*, and *X*_*i*_ are independent of all nondescendant nodes except its parent node set Pa(*X*_*i*_). Therefore, the joint probability distribution of variable set V = {*X*_1_, *X*_2_, ⋯, *X*_*n*_} can be decomposed into

(2) $$\begin{array}{c} \text{P}\left(\text{V}\right)=\text{P}\left(X_{1},X_{2},\cdots ,X_{n}\right)=\overset{n}{\underset{i=1}{\prod }}P\left(X_{i}\;|\;Pa\left(X_{i}\right)\right). \end{array}$$

The Bayesian network model uses a directed acyclic graph to represent the dependent and independent relationship between variables and uses conditional probability distribution to describe the dependent relationship between variables and their parent nodes. Therefore, the establishment of the Bayesian network model includes two parts: (1) determining the relationship between variables to find the network structure, namely, structure learning and (2) determining the conditional probability table of each node, namely parameter learning.

#### 2.3.4. Structural Learning Methods

The MMHC algorithm is used to learn the structure of the Bayesian network. This algorithm combines the methods of dependency analysis and score search and is divided into two stages. The first stage is learning. In this stage, the MMPC algorithm is used to determine each node's candidate parent-child node set, and the undirected framework of Bayesian network structure is constructed. In the second stage, the greedy mountain climbing algorithm is used to search and score the framework of the network structure obtained and find the network structure which makes the scoring function the largest.

The MMPC algorithm uses the max-min heuristic strategy to determine the candidate parents and children (CPC) set of the target variable (T) from the given data set, which is divided into two stages. In the first stage, we define a correlation function to determine the conditional dependence of other variables and target variable *T* under a given CPC. The larger the function value indicates, the stronger the conditional dependence between variables; when the function value is zero, there is no dependency between variables: the independent piece. The max-min heuristic strategy selects the variable with the max-min relevance to the target variable t under the given CPC condition to enter the CPC. When all variables except the variables in the CPC are conditionally independent of the target variable *T* under the given CPC condition, the first stage stops. In the second stage, the variables in the candidate parent-child node-set CPC are tested, and wrong variables are removed. For the variable *X* in CPC, if there is a subset *S* of CPC such that Assoc (*X*, *T*,| *S*), then the variable *X* is removed from CPC.

The correlation function of variables *X* and *T* under given variable set *Z* is defined as

(3) $$\begin{array}{c} \text{Assoc}\left(\text{X},\text{T}\;|\;\text{Z}\right)=2\underset{a,b,c}{\sum }N_{ijk}^{abc}\ln\frac{N_{ijk}^{abc}N_{k}^{c}}{N_{ik}^{ac}N_{jk}^{bc}}, \end{array}$$

where *N*_*ijk*_^*abc*^ is the number of samples satisfying *X* = *a*,*T* = *h*, and *Z* = *c* in data set *D*. The corresponding minimum correlation function is defined as

(4) MinAssocX,T, ∣ Z=AssocX,T ∣ SS⊆Zmin,

where *S* is a subset of variable set *Z*.

### 2.4. Treatment Methods

The 40 patients in the validate database were predicted by the above MMHC algorithm. Among them, 20 cases predicted better curative effect and was defined as the research group. Another 20 patients with poor prognosis were defined as the control group. There was no significant difference in gender, age, TNM stage, tumor type, and follow-up time between the two groups (*P* > 0.05).

Both groups were given pemetrexed disodium (Qilu Pharmaceutical Co., Ltd.) by intravenous drip of 500 mg/m^2^, 10 min/time, for 21 days for 1 treatment cycle. Prophylactic medication was as follows: 7 days before pemetrexed disodium infusion, folic acid 400 g/d was taken orally for 28 days, until the end of pemetrexed treatment. Intramuscular injection of vitamin B12 at 1 000 g/d 7 days before pemetrexed was performed at an interval of 9 weeks. Dexamethasone 4 mg was taken orally for 2 times per day before and after pemetrexed, respectively. CT examination was performed once every 2 cycles of chemotherapy to evaluate the efficacy, and chemotherapy was continued without tumor deterioration or severe adverse reactions. As the tumor worsens, the chemotherapy regimen is changed. Before chemotherapy, patients were given a 5-HT3 receptor antagonist to prevent vomiting, and on this basis, taking anlotinib hydrochloride capsule (Chia Tai Tianqing Pharmaceutical Group Co., Ltd.) orally once per day, with the initial dose of 12 mg/time. The regimen was taken orally before breakfast for 14 d consecutively, with 7 d withdrawal and 21 d as a cycle. If severe toxicity occurred during treatment, the dose of anlotinib was reduced to 10 mg/d or 8 mg/d.

### 2.5. Intelligent Image Segmentation and Diameter Measurement

After the tumor was segmented by artificial neural network, the long diameter of primary tumor and most extensive metastatic lesion was measured to compare the changes between two groups.

#### 2.5.1. Image Preprocessing

CT image is polluted by noise and the image quality decreases. Wiener filter is a classical linear denoising filter. It is often used to recover useful signals from additive noise. It is a filtering method that combines degradation function and noise statistical characteristics. At the same time, the imprecise and fuzzy information of CT image are processed by fuzzy enhancement to enhance the image contrast.

#### 2.5.2. Image Texture Feature Extraction

Texture is a visual feature that reflects the homogeneous phenomenon in the image and reflects the surface structure, organization, and arrangement attribute of the object surface that changes slowly or periodically. Because texture features can provide unique spatial diversity information of regional pixels, it is easy to distinguish between target and background, which is suitable for lung cancer lesion extraction. There are three salient features extracted in this study, namely, image inertia, mean, and entropy, which are obtained from formulas (5)–(7):

(5) $$\begin{array}{c} {tf}_{1}=\overset{N}{\underset{i=1}{\sum }}\overset{N}{\underset{j=1}{\sum }}\left(i-j\right)\times p{\left(i,j\right)}^{2}, \end{array}$$

(6) $$\begin{array}{c} {tf}_{8}=\overset{N}{\underset{i=1}{\sum }}\overset{N}{\underset{j=1}{\sum }}\frac{p\left(i,j\right)}{M\times N}, \end{array}$$

(7) $$\begin{array}{c} {tf}_{10}=\overset{N}{\underset{i=1}{\sum }}\overset{N}{\underset{j=1}{\sum }}\left(i-j\right)\times p\left(i,j\right)\times \mathrm{lg}\left[p\left(i,j\right)\right]. \end{array}$$

#### 2.5.3. Image Fractal Feature Extraction

Fractal feature is used to describe complex and irregular medical image features. Fractal dimension is an important parameter to describe the complexity, irregularity, and spatial distribution trend of nonlinear image, which is calculated by difference box dimension.

The specific steps are as follows: divide the *N* × *N* image into *s* × *s*  blocks. 2 < *s* < *N*/2, let *r* = *n*/*s*, each block contains a column *s* × *s* × *h* of boxes, and *H* is the height of a single box. A 5 × 5 window is used to slide on the image with a moving range of *r*. assuming that the maximum gray value and the minimum gray value in the (*i*, *j*)-th block fall in the *K* and *l* boxes, respectively, the number of boxes required to cover the (*i*, *j*)-th block is calculated by formula (8), and the number of boxes required to cover the whole image is given by formula (9). At this time, the corresponding fractal dimension FD is given by formula (10). Select a group of *S*, and the fractal dimension FD can be obtained by linear fitting:

(8) $$\begin{array}{c} n_{r}\left(i,j\right)=l-k+1, \end{array}$$

(9) $$\begin{array}{c} N\left(r\right)=\underset{i,j}{\sum }n_{r}\left(i,j\right), \end{array}$$

(10) $$\begin{array}{c} \text{PD}=\frac{\log\left[N\left(r\right)\right]}{\log\left(1/r\right)}. \end{array}$$

#### 2.5.4. Artificial Neural Network

Artificial neural network has the ability of self-learning and self-adaptive. It can determine the potential law between the two by pretraining samples and prediction samples and calculate the new input sample data by using the rules formed in the training stage.

When using ANN to segment the image, all points in the image to be segmented are clustered into target and nontarget pixels, and the nontarget pixels are removed after accurate clustering, so as to obtain the target image. The specific steps are as follows.

1. A *c*-layer neural network is set. For example, the input mode *P* is added to the input layer, the sum of *y* unit inputs in layer *z* is *U*_*x*_^*z*^, the output is *U*_*j*_^*k*^, and the combination weight from the *j*-th neuron in layer *z* − 1 to the *x*-th neuron in layer *z* is *W*_*xy*_. If the relationship function between input and output of each neuron is *f*, the relationship between variables is shown in formulas (11)–(13):

(11) $$\begin{array}{c} V_{x}^{z}=f\left(U_{x}^{z}\right), \end{array}$$

(12) $$\begin{array}{c} U_{x}^{z}=\underset{y}{\sum }W_{xy}V_{x}^{z-1}, \end{array}$$

(13) $$\begin{array}{c} \text{f}\left(\text{h}\right)=\frac{1}{1+e^{-h}}. \end{array}$$

(2) Define the error function *E* as the square sum of the difference between the expected output and the actual output, as shown in the formula (14). The ANN learning process is to find the minimum value of the error function. The gradient descent method of nonlinear programming is used to obtain the update ∆*W*_*y*_^*x*^ of the weight *W*_*y*_^*x*^, as shown in the formula (15). *ε* is the learning rate, with a value of 0-1:

(14) $$\begin{array}{c} \text{E}=\frac{1}{2}\underset{y}{\sum }{\left(V_{y}^{c}-T_{y}\right)}^{2}, \end{array}$$

(15) $$\begin{array}{c} ∆W_{y}^{x}=-\varepsilon \frac{\vartheta E}{\vartheta W_{xy}}. \end{array}$$

(3) After more complex derivation operation, the modified weight is obtained. See the formulas (16) and (17) to complete the convergence of the algorithm:

(16) $$\begin{array}{c} W_{xy}^{`}=W_{xy}-\varepsilon d_{y}^{z}V_{y}^{z-1}, \end{array}$$

(17) $$\begin{array}{c} d_{y}^{z}=V_{y}^{z}\left(1-V_{y}^{z}\right)\underset{p}{\sum }W_{xp}d_{y}^{z+1}. \end{array}$$

In order to avoid over fitting, the formula (18) is used to obtain the upper limit of the number of hidden layers *N*_*h*_, where *N*_*i*_ represents the number of neurons in the input layer, *N*_*o*_ represents the number of neurons in the output layer, *N*_*s*_ represents the number of training samples, the value range of *α* is 2-10, and the average value of input and output is used as the lower limit of the hidden layer:

(18) $$\begin{array}{c} N_{h}=\frac{N_{s}}{\alpha \left(N_{i}+N_{o}\right)}. \end{array}$$

### 2.6. Criteria for Clinical Efficacy

Patients were followed up until disease progression or intolerance. The RECIST was applied to evaluate the tumor regression of primary tumor after chemotherapy. Complete remission (CR) was as follows: all target lesions are undetectable and duration not less than four weeks. Partial remission (PR) was as follows: compared with the baseline level, the sum of the two diameters of all target lesions is reduced by more than 30%. Progression disease (PD) was as follows: baseline lesion long diameter increased not less than 20% or new lesions appeared. Stable disease (SD) was as follows: sum of the length of the long diameter of baseline lesions did not reach PR or increase did not reach PD:

(19) $$\begin{array}{c} \text{Disease control rate }\left(\text{DCR}\right)=\left(\text{CR}+\text{PR}+\text{SD}\right)/\text{total cases}, \end{array}$$

(20) $$\begin{array}{c} \text{Objective response rate }\left(\text{ORR}\right)=\left(\text{CR}+\text{PR}\right)/\text{total cases}, \end{array}$$

which compared the progress free survival (PFS) between them after treatment.

### 2.7. Statistical Methods

Use SPSS 20.0 statistical software. The measurement data were measured by mean ± standard deviation, and the count data was described by component ratio or rate (%) and using *χ*^2^ test for comparison between groups.

## 3. Results

### 3.1. Intelligent Image Segmentation Results

The image preprocessing results are shown in Figure 1, in which Wiener filtering eliminates image noise, and the image contrast is significantly improved after fuzzy enhancement.

### 3.2. Measurement of the Maximum Diameter of Solid Tumor Lesions

After two courses of treatment, the maximum diameter of primary foci and metastatic foci in both groups was significantly reduced compared with that before treatment (Figure 2). The solid tumors in the research group shrank significantly, surpassing the control group. The difference was statistically significant (*P* < 0.05, Figures 3 and 4). The three-dimensional (3D) reconstruction results from the segmented images showed that the tumor volume in the research group was significantly reduced than in the control group (Figure 5).

### 3.3. Comparison of Clinical Efficacy between Two Groups

After treatment, the ORR and DCR of the control group were 20.0% and 75.0%; the ORR and DCR of the research group were 20.0% and 90.0%, respectively; the DCR of the research group was significantly higher than that of the conventional group (*P* < 0.05), see Table 2.

### 3.4. PFS Comparison between the Two Groups

After treatment, PFS in the research group was 7.1 months, significantly higher than the conventional group (4.8 months). The difference is statistically significant (*P* < 0.01), as shown in Figure 6.

## 4. Discussion

For patients with early NSCLC, surgical treatment is still the primary treatment, but the treatment of advanced NSCLC is still dominated by traditional radiotherapy and chemotherapy. However, with the in-depth research on the EGFR signaling pathway, a series of targeted drugs have been found, and corresponding targeted therapeutic drugs have been developed [16]. At present, the treatment of lung cancer has been upgraded to the level of molecular targeted therapy. The emergence of targeted drugs has prolonged the survival time of NSCLC patients, especially for patients with favorable EGFR mutations and ROS1 and ALK-positive patients, and improved the patients' clinical prognosis and life quality. The clinical efficacy of negative patients without modifications is still low, and there is also a phenomenon of targeted drug resistance in clinical. There is no unified treatment plan in clinical, and the effectiveness of ROS1 drug treatment is quite different [17]. Therefore, the development of new targeted therapeutic drugs has become a hot issue in this field.

Anlotinib can inhibit VEGF1, 2 ,and 3, *α* and *β*, platelet-derived growth factor receptor, fibroblast cell growth factor receptors-1, 2, 3, and 4, C-kit, and other targets. This drug plays a robust inhibitory effect and then plays a role in inhibiting tumor blood vessel growth and tumor growth [18, 19]. Related studies have found that anlotinib has certain advantages in the clinical efficacy and safety of treating patients with NSCLC. It can provide new therapies for refractory NSCLC patients who have failed multiline chemotherapy and drug resistance [20]. Pemetrexed is an antimetabolic drug that can block purine and pyrimidine synthase, thereby preventing cell proliferation and playing an antitumor effect. Pemetrexed has a good impact on various tumors, especially NSCLC and malignant mesothelioma [21, 22].

In this study, it was found that the DCR of anlotinib hydrochloride combined with pemetrexed could be effectively improved and prolong the PFS of the patients. After treatment, the patient's daily life, emotional control, activities, social/family life, and other scores were higher than before treatment, and the total score was also higher than before treatment. The results indicated that combined treatment has certain advantages in clinical efficacy and safety in treating patients with NSCLC. The consideration may be related to the following reasons. Firstly, anlotinib acts as a tumor suppressant through targeted inhibition of angiogenesis and cell proliferation-related kinases. Secondly, by using molecular targeting to treat patients with NSCLC, the body damage caused by chemotherapy is avoided, and the life quality of patients can be improved [23]. This study also found that combined treatment can increase the incidence of hand-foot syndrome in patients. Therefore, when using anlotinib to treat patients, attention should be paid to complications such as hand-foot syndrome to avoid serious consequences.

The development of targeted drugs is expensive, which brings a severe economic burden to patients. If the curative effect is not exact, it is not worth the loss for the whole family. Therefore, the ideal way is to evaluate the prognosis of patients in advance. If the prognosis is good, the use of drugs is more reasonable. Based on the data collected in the past five years, this study established a prediction model using the MMHC algorithm. Then, we make a further prospective study using this model. Under the guidance of the model, the research group has a lower diameter of primary foci and metastatic foci, a higher ORR, DCR, and a longer PFS than the control group. The results further confirm the role of the MMHC algorithm in the precise treatment of NSCLC. In addition, many factors may influence the prognosis, mainly the histological grade, tumor stage, diagnosis age, tumor size, number of examined lymph nodes, and number of positive lymph nodes. The MMHC algorithm model is the result of a comprehensive analysis.

## 5. Conclusions

In summary, under the guidance of the MMHC algorithm modes, the combination of Anlotinib hydrochloride capsules and pemetrexed disodium chemotherapy in the treatment of advanced NSCLC is more effective, which is conducive to the prognosis judgment and treatment cost control. There are some shortcomings in this study. The sample of patients was small, which needs to be further improved in the future. In the future, we will apply more algorithms to predict the efficacy of drugs.

## Figures and Tables

**Figure 1:** Image preprocessing of lung cancer. (a)–(c) gray image. (d)–(f) Wiener filtering. (g)–(i) Fuzzy enhancement.

**Figure 2:** CT observation before and after treatment in the two groups. (a) Control group before treatment. (b) Control group after treatment. (c) Research group before treatment. (d) Research group after treatment.

**Figure 3:** Comparison of maximum diameter of the primary lesion between the two groups before and after treatment. ^∗^Compared with the data before treatment, *P* < 0.05; ^∗∗^compared with the data before treatment, *P* < 0.01.

**Figure 4:** Comparison of maximum diameter of the largest metastases between the two groups before and after treatment. ^∗∗^Compared with the data before treatment, *P* < 0.01.

**Figure 5:** Three-dimensional reconstruction before and after treatment in the two groups. (a) Control group before treatment. (b) Control group after treatment. In the control group, the tumor volume decreased from 53.6 cm^3^ to 48.1 cm^3^ (5.5 cm^3^). (c) Research group before treatment. (d) Research group after treatment. In the research group, the normal lung volume increased from 2139.0 cm^3^ to 2327.4 cm^3^, equivalent to the reduction of tumor volume by 188.4 cm^3^.

**Figure 6:** Progression-free survival curves for the two groups.

**Table 1:** Final characteristic variables filtered by logistic regression analysis.

Variable	*B*	Std. error	*P*	Exp	95% exp	
Histological grade	—	—	0.002	—	—	—
Tumor stage	—	—	0.011	—	—	—
Diagnosis age	0.058	0.012	0.001	0.931	0.921	0.962
Tumor size	0.015	0.006	0.012	0.978	0.962	0.989
Number of examined lymph nodes	0.048	0.013	0.003	1.049	1.013	1.084
Number of positive lymph nodes	0.187	0.062	0.004	0.821	0.731	0.947

**Table 2:** Comparison of clinical efficacy between two groups of patients.

Group	*n*	CR/case	PR/case	SD/case	PD/case	ORR/%	DCR/%
Control group	20	0	4	11	5	20.0	75.0
Research group	20	0	4	14	2	20.0	90.0^∗^

^∗^ *P* < 0.05 vs. conventional group.

## Data Availability

The data used to support the findings of this study are available from the corresponding author upon request.
